The article "Discuss the Application of Data Services in Data Health Management of High-Risk Pregnant and Lying-In Women in Smart Medical Care" was retracted in 2023. Reasons: signs of a paper mill; suspected computer-generated content; unreliable results or conclusions; lack of ethics approval or compliance.

# Discuss the Application of Data Services in Data Health Management of High-Risk Pregnant and Lying-In Women in Smart Medical Care

**DOI:** 10.1155/2022/5957697

**Published:** 2022-08-25

**Authors:** Leifen Shen, Weiqin Shi, Liwen Cai, Jing An, Qian Ling

**Affiliations:** ^1^Maternity Group Healthcare Department, Huzhou Maternity & Child Health Care Hospital, Huzhou, Zhejiang 313000, China; ^2^Healthcare Department, Huzhou Maternity & Child Health Care Hospital, Huzhou, Zhejiang 313000, China; ^3^Child Group Health Department, Huzhou Maternity & Child Health Care Hospital, Huzhou, Zhejiang 313000, China; ^4^Obstetrics and Gynecology Department, Huzhou Maternity & Child Health Care Hospital, Huzhou, Zhejiang 313000, China

## Abstract

**Objective:**

In order to improve the refined management of hospitals, promote the scientific development of smart hospitals in medical institutions, and solve the problem of data filling and reporting that is increasing year by year in the country, province, and city.

**Methods:**

A total of 84 high-risk pregnant women admitted to our hospital from January 2020 to October 2021 were selected and screened for high-risk pregnant women. Risk pregnant women were divided into a routine intervention group and a DS medical group, with 42 cases in each group. High-risk pregnant women in the routine intervention group received routine intervention, and the DS medical group applied data to serve smart medical services on the basis of routine intervention. The scores of self-care, anxiety, and depression were compared between the two groups, the coping styles were analyzed, the satisfaction rate and incidence of adverse conditions of the high-risk puerperae were recorded, and the delivery methods of the two groups were compared.

**Results:**

After the intervention, the activities of daily living, follow-up, fetal monitoring, and self-protection behaviors in the DS medical group were higher than those in the routine intervention group, and the difference was statistically significant (*P* < 0.05). The scores of anxiety and depression in the group were lower, with statistical significance (*P* < 0.05); after the intervention, the scores of negative coping styles in the DS medical group were lower than those in the conventional intervention group, while the scores for positive coping styles were higher than those in the conventional intervention group; the DS medical group had higher risk. The satisfaction of pregnant women was significantly higher than that of the routine intervention group, and the difference was statistically significant (*P* < 0.05); the overall incidence of adverse maternal outcomes among high-risk pregnant women in the DS medical group was lower than that of the routine intervention group, and the difference was not statistically significant (*P* > 0.05). Compared with the routine group, the DS medical group had a higher number of vaginal deliveries and a lower number of cesarean deliveries, and the difference was statistically significant (*P* < 0.05).

**Conclusion:**

The application of data services in a smart medical high-risk maternity-related data management platform enables the promotion of high-risk pregnant women's self-care behaviors and improves negative emotions, enables them to cooperate in delivery with positive behaviors, and reduces the number of cases of cesarean delivery.

## 1. Introduction

High-risk pregnant women have a high risk of dystocia and preterm delivery, which may lead to a series of postpartum complications in serious cases [1, 2]. Effective nursing intervention is conducive to reducing maternal mortality, which makes it of great significance to grasp the health status of high-risk pregnant women [3]. With the progress of medical technology, data services have been effectively and widely applied [4]. In the context of the rapid formation of smart medical services, it is necessary to pay timely attention to high-risk pregnant women through data analysis in order to strengthen the protection of themselves and their fetuses [5]. Data services: data extraction based on smart medicine, referred to as DS system platform, provides support for hospital management capabilities through the application of data technology and intelligent means [6]. In order to provide basis for the construction of high-level intelligent hospitals with data-driven core, this paper chooses to explore the application of data services in the intelligent medical data management platform for high-risk pregnant women, so as to provide support for strengthening the core competitiveness of hospitals.

## 2. Materials and Methods

### 2.1. Material

A total of 84 high-risk pregnant women treated in our hospital from January 2020 to October 2021 were selected. High-risk pregnant women were divided into the routine intervention group and the DS medical group, 42 cases in each group. The age of the conventional intervention group was 22 to 42 years old, with an average age of 31.95 ± 9.84 years and an average gestational age of 38.99 ± 1.26 weeks. There were 39 primiparas and 3 multiparas. The age of the DS group ranged from 23 to 44 years old, with an average age of 32.56 years (10.74 years) and an average gestational age of 38.93 weeks (1.22 weeks). There were 40 primiparas and 2 multiparas. There was no statistical difference in the general data of high-risk pregnant women between the two groups (*P* > 0.05), indicating comparability.

Inclusion criteria are as follows: ① the data were complete, all were single pregnancy, ② including bleeding during pregnancy, pregnancy complications, and abnormal pregnancy history.

Exclusion criteria are as follows: ① heart, lung, and liver dysfunction; ② diabetes history; ③ people with mental illness; ④ data not complete; (5) multiple children; ⑥ poor compliance; and ⑦ the existence of immune diseases.

### 2.2. Methods

#### 2.2.1. Intervention Methods

In the routine intervention group, high-risk pregnant women were treated with traditional management mode and examined before delivery. Medical staff for pregnancy guidance and psychological intervention pay close attention to maternal blood pressure, blood sugar, and other levels. The medical staff observed the progress of puerpera's labor and assisted puerpera's delivery.

On the basis of the routine intervention group, the DS medical group applied data services to intelligent medical services. First, the DS medical team was established, consisting of doctors, midwives, and obstetric nurses. Develop manuals on integrated medical, nursing, and patient services. And train team members to master work procedures and standards. Quasidiagnostic services were as follows: examination and evaluation, health education, health education files, physiological status nutrition, weight management, healthcare of physiological status, skull defect screening, common discomfort treatment, skull education, and skull observation. The data were recorded, and the risk of pregnancy was assessed. Data extracted from data services is used to establish background database on the basis of intelligent medical treatment, so as to facilitate the guidance of nursing intervention for high-risk pregnant women by medical staff. The medical team collected data on the conditions of pregnant women during the nursing process. After the data is uploaded to the platform through DS, it will be analyzed by doctors and then medical intervention will be carried out. Through data service intelligent medical data analysis of high-risk maternal psychological status, psychological care is given. In particular, for older pregnant women, nursing staff should timely communicate with pregnant women and give them psychological comfort to promote their elimination of psychological barriers and build confidence in treatment. Throughout the labor: once the woman is in labor, the team achievement collects data and provides ongoing psychological, physical, secular, and physical support and care according to the delivery schedule. Members of the team should work closely to understand the mix of medical treatment and medical assistance. Based on data services, data support to perceive dynamic changes in maternity and analyze treatment plans and events at medical assistance points and implement them. After the establishment of high-risk maternal archives, high-risk maternal risk screening and scoring were performed. Dynamic pregnancy of pregnant women with higher scores was followed; high scores of late pregnant women, for many visits, carefully recorded, ready for delivery at any time. Establish a reasonable plan. At the same time, for high-risk pregnant women, a daily diet and exercise plan should be made. Provide pregnant women with affordable nutrition and acceptable exercise based on relevant risk factors, and specify the amount of exercise.

#### 2.2.2. Self-Care Management Score

The maternal self-care management level questionnaire independently developed by our hospital was used to evaluate and compare the self-care management level of the two groups after intervention and before intervention. Cronbach's *O* coefficient was *L*0.852, and the retest validity was 0.862, covering daily life (8 items). Compliance behavior (4 items), fetal monitoring behavior (5 items), and self-protection behavior were divided into 4 dimensions, with 2 items for each. Each item was graded from 1 to 5 with a score of 25 to 125. There was a positive correlation between the level of self-care management behavior and the evaluation score.

#### 2.2.3. SAS and SDS Scores

In this study, SAS and SDS scores were used to compare the anxiety and depression of high-risk pregnant women. SAS is an anxiety scale with a total score of 100 and 20 items. According to the 4-point scoring method, the higher the score, the more serious the disease. SDS is a scale commonly used in clinical evaluation of inhibition [7]. The total score was 100 points, and there were 20 items. The higher the score, the more serious the disease.

#### 2.2.4. Scoring Coping Style

Summary coping style questionnaire (SCSQ) was used to evaluate coping style of high-risk pregnant women before and after intervention, including 12 items of positive coping style and 8 items of negative coping style. Grades are given on a 4-point scale. When the positive coping score is high, the corresponding negative score is low, indicating that high-risk pregnant women have a positive coping style [8].

#### 2.2.5. Satisfaction, Adverse Conditions, and Delivery Methods

The two groups of high-risk pregnant women were followed up by senior physicians in our hospital, and the satisfaction of the two groups was evaluated, which was divided into relatively satisfied, satisfied, and dissatisfied, satisfaction = relatively satisfied + satisfied/%. At the same time, the adverse conditions of pregnant women in the intervention process were recorded, including neonatal asphyxia, postpartum hemorrhage, and premature delivery, and the delivery methods of the two groups were recorded by the above-mentioned physicians.

### 2.3. Statistical Treatment

Make use of software general SPSS 20.0 statistical data analysis using software operation mode which can sample statistical data analysis and data processing. () was used to compare the measurement error between sample groups, and *t*-difference was used to compare the calculation error of frequency comparison between groups. Measurement data line % inspection. The intergroup mean error: *X*^2^ test was used for the calculation error of intergroup frequency comparison, and *P* < 0.05 indicated statistically significant difference.

## 3. Results

### 3.1. Self-Healthcare Analysis

As shown in Figure 1, the comparison of daily life, compliance with doctors, fetal monitoring, and self-protection behaviors between the two groups before intervention was not statistically significant (*P* > 0.05). After intervention, the daily life, compliance, fetal monitoring, and self-protection behaviors of the DS medical group were higher than those of the conventional intervention group, with statistical significance (*P* < 0.05).

### 3.2. Comparison of Anxiety and Depression Scores

As shown in Figure 2, before intervention, the anxiety scores and depression scores of the two groups were not statistically significant (*P* > 0.05). After intervention, the scores of anxiety and depression in the DS medical group were lower than those in the conventional intervention group, which was statistically significant (*P* < 0.05).

### 3.3. Comparison of Coping Style Scores

As shown in Figure 3, before intervention, there was no statistical significance in the scores of coping styles between the two groups compared with the conventional intervention group (*P* > 0.05). After intervention, the DS group scored lower on negative coping style. The positive coping score was significantly higher than that of the conventional intervention group (*P* < 0.05).

### 3.4. Satisfaction Analysis of the Two Groups

As shown in Table 1, the satisfaction degree of high-risk pregnant women in the DS medical group was significantly higher than that in the routine intervention group, which was statistically significant (*P* < 0.05).

### 3.5. Comparison of Adverse Events

As shown in Table 2, the total incidence of adverse events in high-risk pregnant women in the DS group was lower than that in the routine intervention group, and the comparison between the two groups was not statistically significant (*P* > 0.05).

### 3.6. Comparison of Delivery Methods between the Two Groups of High-Risk Pregnant Women

As shown in Table 3, compared with the conventional group, there were more cases of vaginal delivery and fewer cases of cesarean delivery in the DS medical group, which was statistically significant (*P* < 0.05).

## 4. Discussion

High-risk pregnancy refers to certain complications or pathogenic factors during pregnancy, which may harm pregnant women, fetuses, and newborns or lead to dystocia. Pregnant women with high-risk pregnancy factors are called high-risk pregnant women [9]. Management of high-risk pregnant women is an important link in improving obstetric quality. Timely intervention and screening enable pregnant women to receive corresponding medical services in time according to the situation, which helps reduce the complications of high-risk pregnant women [10, 11]. Healthcare information management is widely used in Europe and America and has achieved remarkable results in clinical application. Therefore, the information management system has been established in most countries [12, 13]. Recording individual medical information in the computer reduces the incidence of medical errors, thus improving the overall level of medical treatment and providing better medical services for patients [14, 15]. The method of DS data extraction is parallelism between system instances and serial extraction of tables between system instances [16]. Compared with other data processing systems, DS has the characteristics of high speed and efficiency in processing big data [17].

Clinical studies have found that high-risk pregnancy will seriously threaten the life and health of the fetus and pregnant women and even cause dystocia and neonatal asphyxia. The main factor leading to the increase in the rate of neonatal defects is that pregnant women do not have regular prenatal checkups. In strengthening the management of high-risk pregnant women, we should consider from various aspects. The mother needs to be protected and the newborn needs to be considered. Strengthen the relevant health knowledge and safety education, and strengthen the awareness of maternal self-protection. Through the support of medical data, pregnant women should be arranged for maternity checkup in a timely manner. In addition, prenatal education should be strengthened to enable pregnant women to have a comprehensive understanding and understanding of themselves and their importance, which can help reduce the occurrence of neonatal defects [18].

The results of this study showed that the application of data services in intelligent medical data management platform combined with routine intervention resulted in higher daily life, compliance with doctors, fetal monitoring, and self-protection behaviors of high-risk pregnant women, indicating that the application of data service intelligent medical data management platform can help promote the self-care of high-risk pregnant women. The reason may be the analysis of high-risk pregnant women based on the data service intelligent medical data management platform, which enables medical staff to guide and intervene high-risk pregnant women in a timely manner, thus promoting the self-care behavior of high-risk pregnant women.

At present, most cities in our country's medical institutions also established medical information management system; the application of this management system is to strengthen and improve the management ability and level of pregnant women themselves, and at the same time, the hospital in-patient department accordingly lowers the danger in pregnant women throughout the pregnancy, thereby reducing the labor cost management of pregnant women [19]. In high-risk pregnant women, timely analysis of maternal status and effective guidance can enable high-risk pregnant women to actively face difficulties [20]. Positive attitude towards the disease and effective cooperation with doctors' guidance can help reduce the risk of high-risk pregnant women [21]. The research results of this paper show that the application of data services in the intelligent medical data management platform for high-risk pregnant women can improve their anxiety, depression, and other negative emotions.

Childbirth is a persistent and intense stress source for puerpera, especially for high-risk pregnant women, which inevitably leads to fear, anxiety, depression, and other negative psychological states of high-risk pregnant women [22]. The relationship between psychological factors and human health and disease rehabilitation has attracted more and more attention [23]. In maternal status, anxiety and depression are psychological problems—kinds of expression form; the mood changes in pregnant women have now been confirmed to cause uterine hypoxia, thus reducing uteroplacental blood flow, and fetal blood anoxia happens, such as during cesarean delivery operation, reducing the degree of tolerance of pregnant women more, the incidence of fetal blood anoxic increases more [24]. The research results of this paper show that the application of data services in the intelligent medical-related data management platform for high-risk pregnant women has a higher positive response score. The application of the data services in data management platform enables high-risk pregnant women to give birth actively.

The risk of maternal death during the perinatal period is strongly linked to maternal age, chronic diseases, pregnancy complications, and bad behavior, which in severe cases can have a significant impact on pregnancy outcomes. Based on this, the level of opportunity for adverse pregnant women was comprehensively assessed. Through different levels of early warning and tracking, effective nursing management is implemented to achieve dynamic health management. It is helpful for timely detection of adverse events and has good application value for the development of puerpera and newborn. The research results of this paper show that the application of data services in the intelligent medical-related data management platform for high-risk pregnant women has a high degree of satisfaction. The number of cases of vaginal delivery was more than that of cesarean section.

In conclusion, the application of data services can promote the self-care behavior of high-risk pregnant women, enable them to cooperate with delivery with positive behavior, and reduce the number of cesarean section cases [25].

## Figures and Tables

**Figure 1:** Comparison of maternal self-care levels between the two groups.

**Figure 2:** Comparison of anxiety and depression scores between the two groups.

**Figure 3:** Comparison of coping style scores between the two groups.

**Table 1:** Comparison of satisfaction between two groups [*n*, %].

Group	Number of cases (*n*)	Very satisfied	Satisfied	Dissatisfied	Satisfaction (%)
Conventional intervention group	42	21 (50.00)	12 (28.57)	9 (21.43)	33 (78.57)
DS medical group	42	24 (57.14)	16 (30.09)	2 (4.76)	40 (95.24)
*x* ^2^					5.126
*P*					0.024

**Table 2:** Comparison of adverse events between the two groups [*n*, %].

Group	Number of cases (*n*)	Neonatal asphyxia	Postpartum hemorrhage	Premature delivery	Overall incidence (%)
Conventional intervention group	42	2 (4.76)	2 (4.76)	3 (7.14)	7 (16.67)
DS medical group	42	1 (2.38)	2 (4.76)	2 (4.76)	5 (11.90)
*x* ^2^					0.389
*P*					0.533

**Table 3:** Comparison of delivery modes between the two groups of high-risk pregnant women [*n*, %].

Group	Number of cases (*n*)	Mode of vaginal delivery	Mode of cesarean delivery
Conventional intervention group	42	25 (4.76)	17 (4.76)
DS medical group	42	34 (2.38)	8 (4.76)
*x* ^2^		6.523	
*P*		0.011	

## Data Availability

The data used to support the findings of this study are available from the corresponding author upon request.
